# Three-Dimensional Biomechanical Finite Element Analysis of Lumbar Disc Herniation in Middle Aged and Elderly

**DOI:** 10.1155/2022/7107702

**Published:** 2022-01-15

**Authors:** Shiyuan Wan, Bin Xue, Yanhao Xiong

**Affiliations:** Department of Orthopaedics and Traumatology of TCM, Ruijin Hospital Affiliated to Medical College of Shanghai Jiaotong University, Shanghai 200025, China

## Abstract

Lumbar intervertebral disc protrusion disease refers to the degeneration of intervertebral disc, rupture of fibrous ring, nucleus pulpous protrusion and stimulation or compression of nerve root. The import command in Mimics medical 3D reconstruction software was used to erase the irrelevant image data and obtain vertebral body images. The original 3D model of each vertebral body was built by 3D computing function. A three-dimensional finite element model was established to analyze the effect of different surgical methods on the mechanical distribution of the spine after disentomb. The stress distribution of the spine, intervertebral disc, and left and right articular cartilage at L4/L5 stage and the position shift of the fourth lumbar vertebra were analyzed under 7 working conditions of vertical, forward flexion, extension, left and right flexion, and left and right rotation. The results showed that the established model was effective, and the smaller the area of posterior laminar decompression was, the lesser the impact on spinal stability was. The PELD treatment of lumbar disc herniation had little impact on spinal biomechanics and could achieve good long-term biomechanical stability. Combining the clinical experiment method and finite element simulation, using the advantages of finite element software to optimize the design function can provide guidance for the design and improvement of medical devices and has important significance for the study of clinical mechanical properties and biomechanics.

## 1. Introduction

Lumbar disc herniation refers to the partial or total rupture of the lumbar disc annulus fibrosis caused by various reasons, in which the nucleus pulpous protrudes backward from the rupture and presents stimulation or compression of nerve roots and caudal equine, which is common among people aged 40–60 years [1]. The aetiology of lumbar disc herniation and its relationship to low back pain and sciatica are not fully understood, but are likely to involve a complex combination of mechanical and biological processes. Only 4 to 6 percent of people with lumbar disc herniation experiences severe symptoms [2]. Surgical intervention in patients with lumbar disc herniation accounts for only 1% to 3% of patients. About 80% of people have experienced some degree of lumbar and leg pain [3, 4]. In quite a number of patients, conservative treatment with physical therapy can relieve pain, and since the disc receives the least pressure during bed rest, it is recommended to rest for up to 1 week and then gradually return to normal activity [5]. Surgery is recommended for patients with no relief of pain after at least 6 weeks of conservative treatment. In order to avoid irreversible changes in the nerve root structure caused by chronic compression, conservative treatment is ineffective and the diagnosis and surgical indications are clear. Percutaneous endoscopic lumbar disentomb (PELD) is a percutaneous transforaminal approach under endoscopic laser discectomy. PELD is the minimally invasive surgery with minimum trauma and good surgical effect [6].

Biomechanics is one of the fringe disciplines of osmotic mechanics, biology, and medicine. It is a discipline that explores biology by applying the theory and methods of mechanical problems. Combining medicine and engineering mechanics, it solves the difficult and miscellaneous diseases of biology in clinical diagnosis. Bone tissue and stress restrict each other. When the bone tissue is stimulated by external force, because of being in a stable equilibrium state, the activity of the orthopedist and the orthoclase in the bone tissue will be in an unbalanced state, and the bone will grow abnormally. As the stress decreases, the orthopaedic stone has a larger composition than the osteopath, which reduces some bone mass and increases the stress. Cao et al. extended the model to a complete moving segment, studied the effect of the facet joint transmission of axial load, and established the finite element model of the lumbar posterior structure [7]. Swanson et al. used Ansys software to build a complete L4-L5 3D finite element model, including ligament, posterior spine structure, vertebral endplate, incompressible nucleus pulpous, and annulus fibrosis, and lumbar facet joint was modelled by 3D intervertebral annulus fibrosis. The modelling method of intervertebral annulus fibrosis was similar to Shiraz-ADL. However, the nonlinear displacement of the disc vertebral unit is characterized by initial geometric nonlinearity rather than material nonlinearity. Based on previous studies on the three-dimensional finite element of the lumbar spine, modelling was mainly based on X-ray, computed tomography (CT), magnetic resonance imaging (MRI) data, and frozen section [8]. Kong et al. use a CT scan geometry input model to establish a complex 3D finite element model. Due to the high contrast between the bone and surrounding soft tissue in CT data, the bone geometry can be accurately described. Meanwhile, CT value has an approximate linear relationship with bone apparent density, which can describe bone material properties more accurately. The finite element model mesh can be directly generated based on CT scan results [9]. This model has a real geometry model and has good consistency with experimental data. Therefore, most of the current studies choose to build models based on CT data. However, the processing of soft tissue models such as muscles and blood vessels cannot be well resolved.

The principle of the finite element method is to divide a complex object into a finite number of small elements that can be analyzed mechanically. The process is to discredit the finite element model and replace the original observation object with the finite element model. Different element types are used to set the material attributes of the finite element model. The finite element model is connected by nodes. The internal displacement, stress, and strain of the model under external force can be obtained by precise mechanical analysis of its structure. The finite element method is a powerful tool to analyze the characteristics of complex structures and components by computer. It is a numerical method to simulate and analyze the behaviour or mechanism of structures or components. With the development of computer software technology, there are some computer-oriented techniques in mechanics that can provide a greater chance of success for spinal biomechanics research. The finite element analysis model not only considers the geometry of the research object but also strictly considers the material properties and load conditions. Currently, there are two biomechanical methods of lumbar spine analysis: one through experiments and the other through the creation of computational models. In vitro experiments using fresh human specimens have inherent limitations [10]. Human spinal specimens are difficult to obtain and often have poor bone quality and therefore are not representative of living individuals. When Shu et al. analyzed bones with complex shapes, loads, and boundary conditions, the finite element method was a very useful tool. Special software can be used to model complex structures, demonstrate detailed biomechanical characteristics of the waist, and provide inherent parameters [11]. Helal and Wang pointed out that bilateral posterior pedicle screws were better than unilateral ones in terms of stability in postoperative flexion by studying different surgical modalities and finite element analysis of the number and mode of internal fixates in transformational antibody fusion [12]. Through the finite element analysis of the influence of the screw position on the load transfer of the lumbar pedicle screw, R. Liang et al. pointed out that the position of the pedicle screw plays a significant role in the stability of the spine. Considering the angle of capital plane and axial plane, it plays a significant role in influencing the risk of screw loosening and screw breakage in vivo [13]. Using finite element analysis and 3D printing reconstruction technology, Ayali and Bilginaylar obtained the 3D model of normal lumbar vertebra, including vertebra, intervertebral disc, and ligament and analyzed the internal stress changes of the spine under compression, extension, and axial rotation load. The finite element analysis results had good biomechanical accuracy and verified the effectiveness of the model [14].

In this article, a 3D finite element model was established with the 3D computing function to analyze the effects of different surgical procedures on the mechanical distribution of the spine after discectomy. The stress distribution of the spine, intervertebral disc, and left and right articular cartilage was analyzed under specific loading conditions.

## 2. Contents and Methods

### 2.1. Research Object

A total of 33 healthy volunteers were selected to take lumbar CT, MRI, and anteroposterial-lateral X-ray in the radiology department of a hospital. Chinese volunteers aged between 25 and 35 years, and patients and their families were informed of the whole process of the study and agreed to accept the finite element analysis. Before the experiment, imaging examinations (CT, MRI, etc.) were performed on the volunteers to support diagnosis, and no obvious abnormalities were found. Patients with cerebrovascular and other serious organic brain diseases were excluded. Patients suffering from serious physical diseases such as hypertension, heart disease, and diabetes were excluded; patients with other liver diseases, infectious diseases, and malignant diseases and tumours were excluded; patients without supported imaging diagnosis (CT, MRI, etc.) were excluded.

### 2.2. Main Experimental Equipment and Software

A Lenovo M490 notebook computer is equipped with Intel Core i-53210MCPU, dual-core four-thread 2.5 GHz processor, NVIDIA GEFORCE720M independent graphics card, 4 GB memory, and 500 GB hard disk. The software used included Mimics medical 3D reconstruction software, Geomagic Studio software, Unigraphics NX, 3D design software, and finite element analysis software Ansys Workbench.

Geomagic Studio is a reverse engineering software from Geomagic, which has the advantages of higher computational efficiency, cleaner operation interface, and automated workflow, as a complement to CAD, CAE, and other software [15]. The software can repair and delete the 3D model well and finally generate a higher quality model. The output files are Standard Template Library (STL), Initial Graphics Exchange Specification (IGES), Computer-Aided Design (CAD), and other file formats. In this study, the software was used to repair the model in order to generate a more accurate finite element model.

### 2.3. CT Data Acquisition

Dual-source CT was used to perform thin-layer scan of the lumbar spine, and 255 2D plane images of the CT section were obtained, which were saved in the DICOM format [16]. Using the import command in Mimics medical 3D reconstruction software from Materialise, the CT image saved in the DICOM format was imported to adjust the threshold value of the image. Mask layers of lumbar 3 to 5 vertebral bodies were made. Erase command in Edit Masks was used to erase irrelevant image data to obtain the vertebral body images we needed. Three-dimensional computing function was used to build original 3D models of each vertebral body and save them in the STL format.

### 2.4. Intervertebral Discs and Ligaments

The disc and ligament are built by an anatomical structure. In Unigraphics NX 3D design software, the starting and ending points of the ligament are determined, the width of the ligament is set, the 3D model of the ligament is obtained by sweeping, the shape of the annular fiber and nucleus pulposus is drawn between the vertebral bodies, and the model entity is obtained by stretching. The disc model was obtained by Boolean operation [17]. The model into finite element analysis software Ansys, according to different materials to choose different grid unit size precision, adopts the method of ten nodes tetrahedron division and the experimental model of different materials with different properties. In this article, we study the basis of grid quality analysis and apply the software to complete the grid analysis tool. This software can be convenient to the spinal model of mechanical loading and constraints, and to obtain the desired results.

### 2.5. Surgical

Bone structure, ligaments, and joints are homogeneous, continuous, and isotropic elastic linear materials. All materials contact closely, the vertebral body contact at the joint surface is a nonlinear friction contact, friction 0.01. Boundary conditions: the upper endplate surface of L3 vertebral body is the loading area, and the lower endplate area of L5 is the completely fixed constraint. In Mimics, Boolean reduction was used to simulate posterior and lateral intervertebral disc and posterior lamina resection. The normal model, PELD model, MED model, small fenestration model, and particular process resection model were defined as five surgical models I, II, III, IV, and V, respectively.

## 3. Construction of 3D Model

### 3.1. Modelling Software

Mimics is a Materialise's interactive medical image control system, which is mainly used in medical tomography image data processing. It is a highly integrated and easy-to-use 3D image generation and processing software [18]. It can obtain data by scanning medical X-ray, CT, MRI, and other images, build 3D models, and then output common CAD, FEA, RP, and other formats. Mimics plays a very important role in the medical field. It can not only make clinical diagnosis and surgical plan, but also simulate the whole process of surgery and reduce the rate of surgical failure. Mimics mainly consists of the following 5 modules: the basic module includes image import, image segmentation, image visualization, image registration, and image measurement. The structure of the control system is shown in Figure 1.

The basic modules of the control system include image import, image segmentation, image visualization, image registration, and image measurement, and this module can provide the axial, coronal, and capital graphs of the original data, which can carry out greyscale threshold, region growth, Boolean operation, and multilayer editing processing of the image. The Mimics FEA module can quickly process scan data and output corresponding file formats for finite element analysis and CFD. Users can create a 3D model from the scanned data to mesh the surface of the 3D model and apply it to finite element analysis. Med CAD module is a bridge connecting topographic image data and CAD, and scanning data can be communicated and transformed with CAD in a two-way interactive form. In order to verify CAD implants, Mimics input STL file format data can be displayed in the view area of 2D or 3D graphics, which is more convenient to adjust the model design. The Mimics STL+ module interconnects Mimics and RP rapid prototyping technologies through triangles in the file format. Binary and interpolation algorithms can guarantee the accuracy of the model. The input formats of Mimics STL module are STL and VRML, and the output formats are slightly more. The STL + module realizes the reduction of triangular slices by matrix reduction and triangular slice reduction, so that the model can be interpolated to achieve the goal of smoothing. RP-Slice module and most RP machines can connect SLICE format, and RP-Slice module can automatically generate the support structure required by the RP model. The RP-Slice module can process large files quickly and ensure high accuracy and resolution. The output file formats are SLI, SLC, and CLI. The surgical simulation module is a platform for clinical surgical simulation application, providing a powerful three-dimensional toolkit for clinical operations such as astronomy, separation, and implantation, which is of great help to the surgical simulation process.

With the rapid development of computer technology, communication technology and network technology, image analysis, and image processing as well as PACS play an increasingly important role in clinical diagnosis, telemedicine, and medical teaching. DICOM3.0 is an important network standard and communication protocol to ensure that PACS becomes a completely open system. This file is usually composed of DICOM headers and DICOM datasets [19]. The DICOM file header contains information about the identification dataset, such as recording the patient's name, image size, layer thickness, layer spacing, and pixel resolution. For image description, DICOM uses the bitmap method, and usually, the gray value image is stored in 16 bits.

Models in Mimics can be exported in a variety of formats; DXF format is a file format supported by AutoCAD. A CDB file is a nonphysical file, but can be imported directly into the ANSI Workbench FEA module, whose models need to be associated with static structural models for subsequent analysis. VRML format is used for desktop virtual reality. The PLY format allows multiple 3D models to be output into a single PLY file, which not only stores the colours of the models, but also allows collared solid models to be printed on a rapid prototyping machine. STL files have two output formats: one is binary STL file and the other is ASCII STL file; there are some differences. The binary model does not process the file, whereas the text mode transforms the data in a certain way. Binary STL has a small storage space but is fast to read, whereas ASCII STL output is easy to read and modify.

### 3.2. Software of Finite Element Analysis

In the subsequent development process, new application fields have been continuously expanded, including medical 3D modelling based on medical images, rapid prototyping, human anatomy measurement analysis, tissue engineering stent gap analysis, and other fields of computer-aided medicine. It can integrate a large number of obtained DICOM-type image files and construct corresponding 3D geometric graphics or grid models from the processed image files. Finally, the output can be saved in other formats according to the needs of users, ensuring mutual compatibility between different software [20]. The Ansys Workbench platform of finite element analysis software is used in this study. Ansys is a very famous large-scale universal finite element analysis software in the world. Three-dimensional software and medical software can be directly converted to docking, with a very powerful functional module. Annoys software is mainly composed of preprocessing module, analysis and calculation module, and postprocessing module. The module structure of the software functional system is shown in Figure 2.

The preprocessing module includes the following three parts: definition of parameters after the establishment of the finite element model—the first is to define the element type, material properties, and real constants. Modelling provides two methods to establish the solid model: one is from top to bottom, in accordance with the order of point, line, plane modelling; and the other is from bottom to top—first establish nodes, connect nodes into units, and finally form finite element model. There are manual grid division and free grid division, which are very powerful, especially suitable for irregular and complex models. The analysis module solves the problem according to the parameters and load dataset by the analysis type. The solution module contains many types of analysis, such as structural statics analysis, dynamic analysis, and multiphysical field coupling analysis. The postprocessing module can observe the calculation results in the postprocessing module after solving the problem. Postprocessing module mainly consists of two parts: POST1 is a general postprocessing module, where you can view the cloud map of stress and strain. POST26 is also a postprocessing module, which can calculate algebraic and calculus operations of curves.

### 3.3. Three-Dimensional Geometry Model Is Established Based on Mimics

CT imaging technology application in the clinical diagnosis of fault has been quite mature; In terms of CT imaging principles, CT uses X-rays to irradiate the human body, thus forming different tissues or organs of gray image contrast map, and then by the relative position of the pathological change, shape and size to determine the condition, sensitive CT of osseous tissue. Firstly, the DICOM files of CT images collected are imported into Mimics software. Appropriate gray threshold is selected to distinguish the bone tissue from the soft tissue, making the boundary of the vertebral body, sacrum, and other parts clearer. After selecting an appropriate gray threshold value, due to the accuracy of image and software processing, it is necessary to segment the obtained images appropriately and erase the adhesion between the images of the 4th lumbar vertebrae and the 5th lumbar vertebrae, and the 5th lumbar vertebrae and the 1st sacral vertebrae, paving the way for the subsequent acquisition of independent lumbar vertebrae and sacral vertebrae. The model quality was selected as the best. The initial 3D model was generated by dividing the lumbar and sacral vertebrae, and the generated initial 3D model was processed smoothly. The processed STL model of the 5th lumbar spine and sacrum is imported into Geomagic Studio software for surface optimization, seamless connection, and more. Use the hole filling tool to fill the holes in the model. After filling, use the mesh doctor tool to optimize the model after filling the holes until the model has no small parts, small channels, small parts, and other items.

### 3.4. 3D Model Meshing and Detail Construction

The constructed IGES model was imported into HyperMesh software for secondary geometric cleaning, and the intervertebral disc model was constructed according to the morphology and structure of intervertebral disc: According to the characteristics of fibber ring, a structure model with three concentric circles arranged in inner, middle, and outer layers was established, and three concentric fibbers inserted into the annulus were established to simulate the elastic colloidal substance in each fibber-board layer [21, 22]. The nucleus pulpous was modelled according to its position behind the disc and its proportion; the lower surface of L5 and the upper surface of S1 were normalized to construct the end plate with a thickness of 0.5 mm toward the corresponding vertebrae, and the complete intervertebral disc model was finally constructed. The cortical bone structure was simulated by the outermost unit of the vertebral body with a thickness of 0.5 mm and chancellors' bone in the rest of the vertebral body. According to the characteristic that the ligament only suffers tension under stress, the Link180 unit was used to simulate, and the ligament was set up according to the thickness and function of the ligament [23]. The Solid185 tetrahedral element is used to mesh the model.

### 3.5. Finite Element Model Validation

During the establishment of the finite element model, whether the biomechanical properties of the spine of the established model and the actual human body are similar or not will directly affect the validity and accuracy of the subsequent calculation because of the existence of mesh division and the linear elastic unit assumption of the uniform human tissue. The finite element model of middle-aged and elderly lumbar disc herniation constructed in this article is obtained from CT scan, so the validity of the model can be verified by comparing the established model with the results of in vitro spinal biomechanical experiments conducted by predecessors. Under 400 N vertical load and 86 N forward and backward shear force respectively applied to the model, the relative displacement of the centre point on the surface of the vertebral body of model L5 was compared with the in vitro spine measurement results of Berkson et al., as shown in Figure 3.

Figure 3 shows that under 400 N vertical load, the spine measurement result in vitro is 0.51 ± 0.24 mm. In vitro measurements of the spine were 0.6 ± 0.24 mm under 86 N forward shear force. In vitro spinal measurements were 0.6 ± 0.29 mm under 86 N backward shear force. Under the action of the same three loads, the data obtained from the finite element model constructed in this experiment all fall within the range of deviation variation of the in vitro experimental results compared with the literature, indicating that the model built this time can be used for the following experimental research. Sensitivity analysis provides a reference for cone design. Sensitivity analysis shows that the elastic colloidal material in each fiber board layer simulates proportionally fit. The nucleus pulposus can be modelled in proportion to its position behind the disc.

### 3.6. Three-Dimensional Biological Finite Element Analysis

Finally, L3∼5 3D finite element biological models are established, including vertebral body, intervertebral disc, ligament, and other structures, divided into a ten-node tetrahedron unit model. Models I, II, III, IV, and V contained 218,999 nodes, 197,864 nodes, 206,731 nodes, 209,885 nodes, and 185,586 nodes, respectively. Models I, II, III, IV, and V were composed of 125666, 116483, 115654, 117822, and 112844 tetrahedral elements, respectively. Through calculation and analysis, the equivalent stress and vertebral displacement of each part of five models under seven loading modes were obtained.

### 3.7. Under Vertical Loading

The equivalent stress of the lumbar 4-5 intervertebral disc is almost equal among the 5 models, but model III is the largest. The equivalent stress of the L4 vertebral body-specific cartilage in the 5 models is left (I > IV > III > II > V) and right (I > V > II > IV > III). The equivalent stress of the lumbar 4 vertebral body was the largest in model III and the smallest in model V. Model V was the largest, models II, III, and IV were basically equal and close to model I. The equivalent stress of the L4-5 intervertebral disc and L4 vertebral body was larger in model III, but the position shift of the L4 vertebral body was the smallest. The equivalent stress of model IV was smaller, and it was the closest to model I, but the displacement was larger. It indicates that under vertical loading, the more facet joints are removed, the more likely they are to be displaced and unstable. On the contrary, the facet joints remain intact. The lesser the lamina and ligament flavor are removed, the more stress the vertebral body and intervertebral disc receive. Therefore, under the condition of vertical loading, the stress received by model IV was the smallest among the four surgical models and was not prone to damage changes. The displacement was basically equal to that of models II and III, whereas model V was the largest and showed no difference in instability. The comparison of inferior effect forces under vertical loading is shown in Figure 4.

### 3.8. Under Vertical Left-Right Rotation Loading

The equivalent stress of lumbar 4-5 disc model IV was the closest to model I, and model II was the largest. The equivalent stress models III and IV of the left particular cartilage of the L4 vertebral body were the closest to model I, and the stress on the right side was larger (IV > III > I > V > II), but the difference was not significant, indicating that the greater the removal of facet joints under vertical left-handed loading, the greater the stress received, and the easier the damage was. The equivalent stress of the fourth lumbar vertebra was the smallest in model II, the same in models I and IV, and the largest in model III, and the difference between models III and V was larger than that of the other models, indicating that the more the posterior structure was removed, the greater the stress received by the left-rotation active vertebra was, and the degeneration was easy to occur. The lumbar 4 vertebra displacement models III and IV were the closest to model I, and the displacement of model V was the largest, and the difference was larger, indicating that under vertical left-handed loading, the more facet joint removal, the more unstable, but there was no direct correlation between posterior lamina and ligament flavor removal.

The equivalent stress model IV of the lumbar 4-5 intervertebral disc was the closest to model I and had the least damage, whereas model V had the largest damage, indicating that the more the damage of particular cartilage, the greater the stress received by the intervertebral disc. The equivalent stress model IV of particular cartilage on the left side of L4 vertebral body was the closest to model I, but the maximum stress was found on the right side (IV > I > V > II > III), indicating that the stress on bilateral facet joints was significantly different under vertical dextral loading. The equivalent stress model IV was the smallest, models I and V were equal, and model II was the largest, indicating that the more the posterior structure was damaged, the greater the stress received by the vertebral body. Model V had the largest displacement, indicating that the smaller the damage of particular cartilage and ligament flavor was, the smaller the probability of displacement was.  Figure 5 shows the comparison of inferior effect forces under vertical left-right rotation loading.

### 3.9. Under Vertical Forward Bending and Extension Loading

The equivalent stress model IV of the LUMBAR 4-5 intervertebral disc was the closest to model I. The equivalent stress of particular cartilage on both sides of L4 vertebral body was basically the same in the five models, but the left side was larger than the right side (I > III > IV > V > II) and the right side (V > III > II > I > IV). The equivalent stress models IV and V were the closest to model I. The lumbar 4 vertebra displacement models III and IV were the closest to model I, and the displacement of model V was the largest. It indicates that the greater the failure of the rear structure under vertical buckling loading, the greater the stress received. The more complete the structure of the joint, the less stress it receives and the more stable it is.

The equivalent stress of lumbar 4-5 intervertebral disc models III and IV was close to that of model I and that of model V was the largest. For the equivalent stress of the specific cartilage on the left side of the L4 vertebral body, model V measured the smallest result and model IV had the largest result, where IV > III > II > I > V. Model IV had the minimum equivalent stress, model II was equal to model V, and model III had the maximum stress. Model IV had the smallest displacement, and model V had the largest displacement. It indicates that under vertical extension loading, the smaller the damage of the facet joint is, the smaller the stress received is, and the smaller the damage is, the more stable it is.  Figure 6 shows the comparison of inferior effector forces under vertical flexion and extension loading.

### 3.10. Under Vertical Left-Right Load

The equivalent stress of lumbar 4-5 intervertebral disc models III and IV were close to that of model I, and model V was the largest. The equivalent stress of the lumbar 4 vertebral body in model V was the smallest, and that in model I was the largest. Model I had the smallest displacement, model III was the closest to model I, and model V had the largest displacement. This indicates that under vertical left-leaning loading, the greater the facet joint resection, the greater the stress received by the disc, but the vertebral body and the facet joint on the respected side are smaller, whereas the normal facet joint is the opposite. The more the vertebral displacement joint is removed, the larger it is, and vice versa.  Figure 7 shows the comparison of inferior effect forces under vertical left inclining loading.

The equivalent stress of lumbar 4-5 disc model III was smaller and close to that of model I, whereas that of model V was the largest. The equivalent stress of the L4 vertebral body was smaller in models I and IV, and the largest in model V. Model I had the smallest displacement, model III was the closest to model I, and model V had the largest displacement (V > II > IV > III > I). This indicates that under vertical right-leaning loading, the greater the damage of the facet joint, the greater the stress received by the disc. The particular cartilage was the largest on the excised side and the smallest on the intact side. The stress of vertebral body model IV is minimum, indicating that the structure damage is minimum.  Figure 8 shows the comparison of inferior effect forces under vertical right inclining loading.

## 4. Conclusion

The aetiology of lumbar disc herniation and its relationship to low back pain and sciatica are not fully understood, but are likely to involve a complex combination of mechanical and biological processes. In this article, the import command of Mimics medical 3D reconstruction software was used to erase irrelevant image data and obtain vertebral body images. The original 3D model of each vertebral body was established by 3D computing function. The three-dimensional finite element model was established, and the stress concentration of model IV was the smallest in terms of equivalent stress distribution of the lumbar 4-5 intervertebral disc. In terms of the equivalent stress distribution of the fourth lumbar vertebra, the vertical left inclination of model IV was larger than that of model III, and the vertical right inclination of model V was only second to that of model I. From the perspective of the equivalent stress distribution of the left particular cartilage of the fourth lumbar vertebra, the stress distribution of models IV and III was basically similar to that of model I. According to the equivalent stress distribution of the right particular cartilage of the fourth lumbar vertebra, models III and IV avoided left-right rotation activities in the early postoperative period, whereas models III and V avoided left-right roll activities. From the perspective of the position distribution of the fourth lumbar vertebra, facet joint resection is prone to displacement and instability, models III and IV have better advantages in the surgical model, and there is no difference between them. There is still room for improvement of the model by combining the direction of science and the development trend of biomechanics.

## Figures and Tables

**Figure 1:** Structure diagram of the interactive medical image control system.

**Figure 2:** Finite element analysis software functional system module structure diagram.

**Figure 3:** Model calculation results and comparison diagram.

**Figure 4:** Comparison of inferior effect forces under vertical loading.

**Figure 5:** Comparison diagram of inferior effect force under vertical right rotation loading.

**Figure 6:** Contrast diagram of inferior effect force under vertical forward buckling and extension loading.

**Figure 7:** Comparison of inferior effect forces under vertical left incline loading.

**Figure 8:** Comparison of inferior effect forces under vertical right incline loading.

## Data Availability

The data used to support the findings of this study are available from the corresponding author upon request.
